The article "Establishment and External Validation of a Hypoxia-Derived Gene Signature for Robustly Predicting Prognosis and Therapeutic Responses in Glioblastoma Multiforme" was retracted in 2024. Reasons: signs of a paper mill; suspected computer-generated content; unreliable results or conclusions; concerns about the data.

# Establishment and External Validation of a Hypoxia-Derived Gene Signature for Robustly Predicting Prognosis and Therapeutic Responses in Glioblastoma Multiforme

**DOI:** 10.1155/2022/7858477

**Published:** 2022-02-04

**Authors:** Ke Wang, Yang Lu, Zhihong Liu, Min Diao, Lin Yang

**Affiliations:** ^1^Nursing Department, The Second Affiliated Hospital of Shandong First Medical University, Tai'an, 271000 Shandong, China; ^2^Philippine Women's University, 1743 Taft Avenue, 1004 Manila, Philippines; ^3^Neuro Intensive Care Unit, Taian City Central Hospital, Tai'an, 271000 Shandong, China; ^4^Department of Cerebral Hemorrhagic Diseases, Taian City Central Hospital, Tai'an, 271000 Shandong, China; ^5^Pediatric Intensive Care Unit, The Second Affiliated Hospital of Shandong First Medical University, Tai'an, 271000 Shandong, China

## Abstract

**Objective:**

Hypoxia presents a salient feature investigated in most solid tumors that holds key roles in cancer progression, including glioblastoma multiforme (GBM). Here, we aimed to construct a hypoxia-derived gene signature for identifying the high-risk GBM patients to guide adjuvant therapy and precision nursing based on signs of hypoxia.

**Methods:**

We retrospectively analyzed the transcriptome profiling and clinicopathological characteristics of GBM from The Cancer Genome Atlas (TCGA) and Chinese Glioma Genome Atlas (CGGA) cohorts. A series of bioinformatic and machine learning methods were comprehensively applied for establishing a hypoxia-derived gene signature in prediction of overall survival, disease-free survival, disease-specific survival, and progression-free survival. The predictive efficacy of this model was assessed with receiver operator characteristic (ROC) and uni- and multivariate cox regression analysis. The associations of this signature with tumor microenvironment and immunotherapeutic response predictors were evaluated across GBM. RT-qPCR and western blotting were presented for validating the expression of ALDH3B1 and CTSZ in human glioma cell lines (U251, SHG-44, and U87) and normal glial cell line HEB.

**Results:**

Among hallmarks of cancer, hypoxia acted as a prominent risk factor of GBM prognosis. A hypoxia-derived gene signature displayed efficient ability in predicting clinical outcomes. High risk score indicated undesirable prognosis, recurrence, and progression of GBM. Moreover, this risk score displayed positive correlations to immunity and stromal activation. Combining immunotherapeutic response predictors, high-risk patients more benefited from immunotherapy. ALDH3B1 and CTSZ expression had prominent upregulation in glioma cells than normal glial cells.

**Conclusion:**

Collectively, this hypoxia-derived gene signature could become a reliable biomarker for predicting prognosis and therapeutic response and providing theoretical support for hypoxia treatment and precision nursing of GBM patients.

## 1. Introduction

Gliomas represent frequent primary malignancies in the central nervous system [1]. Glioblastoma multiforme (GBM) is a type IV tumor with astrocytic differentiation and the most aggressive and lethal glioma [2]. GBM displays the feature of undesirable clinical outcomes [3]. Patients who develop GBM have the median survival rate of <1 year and high death risks [2]. Numerous studies have developed genomic models for risk stratification and prognosis prediction of GBM [4–6]. Nevertheless, because of technical problems such as limited sample size and individual heterogeneity, most models possess limited reproducibility and none of them have been applied in clinical routine practice.

Hypoxia presents typical microenvironmental characteristics in almost all solid tumors, including GBM [7]. The rapidly proliferative capacity of the tumor exceeds the growth of its surrounding vasculature, causing a 2-9% reduction in normal oxygen level to hypoxia below 2% [8]. There have been numerous reports on the clinical implication of hypoxia in cancer treatment. Hypoxia is a hallmark of the tumor microenvironment that is the local biological environment where solid tumors are located, covering tumor cells and surrounding stromal cells, caused by the imbalance between enhanced oxygen consumption and insufficient oxygen supply [9]. Hypoxia is an independent prognostic factor of human cancers [10]. As tumor cells adapt to hypoxia, they will acquire more aggressive and treatment-resistant cancer phenotypes [11]. Hypoxia may induce alterations in gene expression, which exhibits a critical role in distinct cellular and physiological functions, eventually deteriorating clinical outcomes of patients [12]. An in-depth understanding of hypoxia-relevant genes during cancer development contributes to a breakthrough in cancer immunotherapeutic research as well as offers a theoretical basis for clinical trials to improve therapeutic outcomes and precise nursing of GBM patients with signs of hypoxia.

## 2. Materials and Methods

### 2.1. Data Acquisition and Preprocessing

RNA sequencing profiles (FPKM values) and matched clinical information of GBM were acquired from The Cancer Genome Atlas (TCGA) via the Genomic Data Commons website (https://portal.gdc.cancer.gov/). After removing patients with missing clinical information, 160 GBM patients were included, which were equally separated into training and testing cohorts.  Table 1 listed the clinical features of these patients. Somatic mutation data that were sorted in the form of Mutation Annotation Format (MAF) were also curated from TCGA project, which were analyzed using maftools package [13]. Moreover, we obtained transcriptome data and follow-up information of 657 gliomas from the Chinese Glioma Genome Atlas (CGGA; http://www.cgga.org.cn) which was used as the validation set.

### 2.2. Analysis of Hallmarks of Cancer

The gene sets of hallmarks of cancer were curated from the Molecular Signatures Database (MSigDB; http://www.broadinstitute.org/msigdb) [14]. Based on the expression profiling of the gene sets, these hallmarks of cancer were quantified in GBM samples from TCGA dataset via single-sample gene set enrichment analysis (ssGSEA) of gene set variation analysis (GSVA) package [15]. *Z*-score scaling was used for the ssGSEA score. Univariate cox regression analysis was presented for evaluating the associations of hallmarks of cancer with GBM prognosis.

### 2.3. Weighted Gene Coexpression Network Analysis (WGCNA)

WGCNA package [16] was applied for constructing a scale-free coexpression network according to the expression profiling of GBM samples in TCGA dataset. The genes in the coexpression module that was strongly associated with hypoxia were screened for further analysis.

### 2.4. Construction of a Least Absolute Shrinkage and Selection Operator (LASSO) Prognostic Model

Through survival package [17], univariate cox regression analysis was presented for screening prognosis-related genes in the hypoxia-relevant coexpression module in TCGA dataset. A LASSO prognostic model was then established utilizing glmnet package [4]. Using survival package, risk score was determined in line with the expression value and LASSO regression coefficient of each candidate gene. According to the median risk score, GBM patients were clustered into high- and low-risk groups. Analysis of overall survival (OS), disease-free survival (DFS), disease-specific survival (DSS), and progression-free survival (PFS) was presented in two groups. Time-independent receiver operator characteristic (ROC) curve was depicted for estimating the predictive efficacy of risk score.

### 2.5. Development of a Prognostic Nomogram

Uni- and multivariate cox regression analysis was conducted for screening independent prognostic factors among risk score and clinical features in TCGA dataset. A nomogram model was established through independent prognostic factors with rms package. The performance of the nomogram in prediction of prognosis was evaluated through ROC, calibration curve, and decision curve analysis (DCA).

### 2.6. Functional Enrichment Analysis

Gene set enrichment analysis (GSEA) was applied for investigating pathways associated with risk score through comparison of high- and low-risk groups in TCGA dataset [18]. For each analysis, 1,000 gene set permutations were presented. The top six pathways were put into multiple GSEA gene sets to demonstrate the range of signaling pathways. The gene sets of hallmarks of cancer were set as the reference set. Moreover, the ssGSEA score of hallmarks of cancer in each GBM sample was visualized and compared in high- and low-risk groups.

### 2.7. Estimation of Tumor-Infiltrating Lymphocytes

Estimation of STromal and Immune cells in MAlignant Tumours using Expression data (ESTIMATE; https://sourceforge.net/projects/estimateproject/) [19] was utilized to infer stromal and immune scores that represented stromal and immune cell fractions in GBM samples from TCGA dataset. Through integrating stromal and immune scores, ESTIMATE score was calculated. Cell type Identification By Estimating Relative Subsets Of RNA Transcripts (CIBERSORT) was applied for inferring the abundance levels of 22 immune cells in GBM tissues [20]. Significant results were retained for further analysis.

### 2.8. Quantification of Immune Response Predictors

Cancer immunity cycle covers release of cancer cell antigens (step 1), cancer antigen presentation (step 2), priming and activation (step 3), trafficking of immune cells to tumors (step 4), infiltration of immune cells into tumors (step 5), recognition of cancer cells by T cells (step 6), and killing of cancer cells (step 7) [21]. The activation of the above steps was quantified utilizing ssGSEA in GBM specimens [22]. Immunophenoscore (IPS), an indicator in predicting response to anti-CTLA-4 or anti-PD-1 therapy, was quantified based on MHC-relevant signature, checkpoint or immunomodulator, effector cell as well as suppressor cell [23]. T cell dysfunction and exclusion (TIDE; http://tide.dfci.harvard.edu/) algorithm was calculated to characterize tumor immune evasion mechanism [24]. Tumor mutation burden (TMB) was determined following mutation frequency with number of variants/the length of exons [25]. Limma package [26] was adopted to compare the differences in immune checkpoints and human leukocyte antigen (HLA) genes in high- and low-risk groups.

### 2.9. Prediction of Drug Response

GBM-relevant chemotherapeutic drugs were selected from the Cancer Genome Project (CGP) [27]. The half-maximal inhibitory concentration (IC50) of chemotherapeutic agents was estimated with pRRophetic package [28].

### 2.10. Cell Culture

Human glioma cell lines (U251, SHG-44, and U87) and healthy glial cell line HEB were purchased from American Type Culture Collection (USA), which were maintained in RPMI 1640 medium (HyClone, USA) plus 10% fetal bovine serum (FBS), 100 U/ml penicillin, and 100 *μ*g/ml streptomycin at 37°C in an incubator with 5% CO_2_.

### 2.11. Real-Time Quantitative Reverse Transcription PCR (RT-qPCR)

Total RNA was extracted from cells using Trizol reagent (Beyotime, China). The cDNA was synthesized using cDNA Reverse Transcription Kit (Beyotime, China). The expression of mRNAs was quantified utilizing 7500 Fast Real-Time PCR System and SYBR Green PCR Master Mix. The relative mRNA expression was determined through the 2^-*ΔΔ*Ct^ method with GAPDH as a reference gene.

### 2.12. Western Blotting

The cells were harvested as well as split utilizing RIPA lysate (Millipore, USA). 5 *μ*g protein was separated via 10% SDS-PAGE electrophoresis at 100 V lasting 2 h. Then, protein was electrically transferred onto polyvinylidene fluoride (PVDF) membrane. Under one-hour block through 5% skimmed milk powder at room temperature, the membrane was washed by TBST as well as incubated by primary antibodies against ALDH3B1 (1/1000; ab236673, Abcam, USA), CTSZ (1/1000; ab182575), and Tubulin (1/500; ab6046) overnight at 4°C. Following being washed by TBST, the membrane was incubated by horseradish peroxidase- (HRP-) labeled secondary antibody (1/3000; ab96899) at room temperature lasting 1 h. Afterwards, the membrane was exposed through ECL kit. The gray value of target proteins was quantified utilizing ImageJ software.

### 2.13. Statistical Analysis

Statistical analysis was executed by R (version 4.0.1) as well as GraphPad Prism (version 8.0.1) software. Student's test or Wilcoxon test was utilized for comparison of two groups. The Pearson or Spearman correlation test was used for evaluating the correlations between variables. *P* < 0.05 indicated statistical significance.

## 3. Results

### 3.1. Hypoxia Acts as a Dominant Risk Factor for GBM Prognosis

Through ssGSEA method, this study quantified the activation of hallmarks of cancer across GBM samples in TCGA dataset. Heat map depicted the close associations between hallmarks of cancer in GBM (Figures 1(a) and 1(b)). Univariate cox regression analysis revealed that estrogen response late (*P* = 0.000535), coagulation (*P* = 0.00402), apical junction (*P* = 0.00405), estrogen response early (*P* = 0.0033), angiogenesis (*P* = 0.00527), apical surface (*P* = 0.0105), p53 pathway (*P* = 0.00679), reactive oxygen species pathway (*P* = 0.00992), epithelial-mesenchymal transition (*P* = 0.0182), Kras signaling up (*P* = 0.0176), apoptosis (*P* = 0.0143), UV response up (*P* = 0.0119), glycolysis (*P* = 0.0154), IL2 STAT5 signaling (*P* = 0.0265), complement (*P* = 0.0279), hypoxia (*P* = 0.0261), myogenesis (*P* = 0.0386), TNF*α* signaling via NF*κ*B (*P* = 0.0457), Notch signaling (*P* = 0.0401), xenobiotic metabolism (*P* = 0.0377), Kras signaling down (*P* = 0.0403), and IL6-JAK-STAT3 signaling (*P* = 0.0482) exhibited significant correlations to GBM prognosis (Figure 1(c)). This study further focused on hypoxia during GBM progression. GBM patients were equally clustered into high and low *Z*-score of hypoxia groups. In Figure 1(d), patients with low hypoxia score displayed survival advantage. The top 5000 genes were used for WGCNA across 168 samples. Clustering analysis uncovered that there was no outlier sample (Figure 1(e)). Based on scale independence and mean connectivity, the network was scale-free when power value = 5 and *R*^2^ = 0.837 (Figure 1(f)). Afterwards, 13 coexpression modules were merged (Figure 1(g)). Among them, blue module exhibited the most significant correlation to hypoxia (Figure 1(h)). Moreover, the blue module had the highest gene significance (Figure 1(i)). Therefore, genes in the blue module were linked with hypoxia.

### 3.2. Development of a Hypoxia-Derived Risk Score for GBM Prognosis

Among 271 genes in the blue coexpression module, univariate cox regression analysis uncovered that 23 genes with *P* < 0.05 displayed marked associations with GBM prognosis (Table 2). Through LASSO analysis, genes with regression coefficients not equal to 0 were screened as candidate variables, with the minimum *λ* of 0.1273 (Figure 2(a)). Hypoxia-derived risk score was developed following the following formula: risk score = ALDH3B1 expression∗0.00694744659450728 + CTSZ expression∗7.56792091910429*e* − 05 (Figure 2(b)). Two candidate variables ALDH3B1 and CTSZ were significantly correlated to GBM prognosis (Figure 2(c)). Heat map visualized the prominently increased mRNA expression of ALDH3B1 and CTSZ in the high- than low-risk group (Figure 2(d)). Moreover, ALDH3B1 and CTSZ expression displayed distinct upregulation in GBM than normal specimens (Figures 2(e) and 2(f)). In line with the median value, we separate patients into high- and low-risk groups (Figure 2(g)). There were more patients with dead or recurred status in the high- than low-risk group (Figures 2(h) and 2(i)).

### 3.3. Hypoxia-Derived Risk Score Predicts GBM Prognosis, Recurrence, and Progression

We equally separated patients in TCGA dataset into training and testing sets. We observed that high-risk patients prominently exhibited unfavorable OS in comparison to low-risk patients in the training, testing, and entire sets (Figures 3(a)–3(c)). ROC curves demonstrated that area under the curve (AUC) values of 6-year survival were separately 0.796, 0.827, and 0.86 in the training, testing, and entire sets, confirming the favorable prediction ability of hypoxia-derived risk score for GBM prognosis (Figures 3(d)–3(f)). Moreover, we observed the markedly unfavorable DFS, DSS, and PFS in high-risk patients (Figures 3(g)–3(i)). The above data demonstrated that hypoxia-derived risk score possessed the potential in predicting GBM prognosis, recurrence, and progression.

### 3.4. Hypoxia-Derived Risk Score Acts as a Robust and Independent Risk Factor for GBM Prognosis

We externally verified the efficacy of hypoxia-derived risk score in prediction of OS in the CGGA dataset. With the same formula, we calculated the risk score of each patient. As expected, high-risk patients had prominently poorer OS than low-risk patients (Figure 4(a)). ROC curves showed that AUC values of 3-, 4-, and 5-year survival were separately 0.6, 0.611, and 0.609, indicative of the well prediction ability of this risk score (Figure 4(b)). In comparison to age, sex, and tumor purity, hypoxia-derived risk score possessed a significant advantage in predicting long-term prognosis (Figure 4(c)). Uni- and multivariate cox regression analysis suggested that age and hypoxia-derived risk score served as independent prognostic factors in GBM (Figures 4(d) and 4(e)). In Figure 4(f), this risk score displayed a positive correlation to age. Female patients possessed increased risk score than male patients (Figure 4(g)). A negative association of risk score with tumor purity was found across GBM patients (Figure 4(h)). After stratifying age and risk score, we presented survival analysis across subgroups. We observed that elder and high-risk patients displayed the poorest OS (Figure 4(i)). Nevertheless, no significant differences in OS were found in different subgroups stratified by risk score with sex or tumor purity (Figures 4(j) and 4(k)). Collectively, hypoxia-derived risk score acted as a robust and independent risk factor for GBM prognosis.

### 3.5. Construction of a Prognostic Nomogram in GBM

Uni- and multivariate cox regression analysis uncovered that hypoxia-derived risk score and age acted as independent prognostic factors of GBM (Figures 5(a) and 5(b)). Based on the two independent prognostic factors, we developed a prognostic nomogram for GBM (Figure 5(c)). In line with the median value, we clustered GBM patients into high and low nomogram risk groups. Our data demonstrated that patients with high nomogram risk markedly exhibited poorer OS than those with low nomogram risk (Figure 5(d)). ROC curve was conducted for evaluation of the predictive performance of this nomogram in GBM prognosis. As a result, the AUC of 6 years was 0.862, demonstrating that the nomogram possessed the excellent predictive efficacy (Figure 5(e)). We further verified the nomogram in the CGGA dataset. Consistently, patients with high nomogram risk had prominently worse OS in comparison to those with low nomogram risk (Figure 5(f)). Also, the AUC of 6 years was 0.624, which confirmed the well predictive efficacy of this nomogram (Figure 5(g)). Calibration curve revealed the high consistency between nomogram-estimated and observed OS in GBM (Figure 5(h)). Moreover, GBM patients could benefit from the nomogram prediction (Figure 5(i)).

### 3.6. Association of Hypoxia-Derived Risk Score with Hallmarks of Cancer

GSEA results demonstrated that IL6-JAK-STAT3 signaling, inflammatory response, and complement were positively correlated to hypoxia-derived risk score while Wnt/beta-catenin signaling, E2F targets, and MYC targets were negatively associated with hypoxia-derived risk score (Figure 6(a)). Moreover, this study quantified the activation of hallmarks of cancer across GBM. In comparison to the low-risk group, angiogenesis and epithelial-mesenchymal transition exhibited significantly increased activation in the high-risk group. Meanwhile, marked reduction in the activation of cholesterol homeostasis, interferon alpha response, interferon gamma response, Notch signaling, oxidative phosphorylation, UV response, and Wnt/beta-catenin signaling was found in the high-risk group (Figures 6(b) and 6(c)).

### 3.7. Association of Hypoxia-Derived Risk Score with Tumor Microenvironment of GBM

Through ESTIMATE method, we inferred the overall infiltration levels of immune cells and stromal cells in GBM tissues. In comparison to the low-risk group, there were markedly increased immune score, stromal score, and ESTIMATE score in the high-risk group (Figures 7(a)–7(c)). The abundance of 22 tumor-infiltrating lymphocytes was quantified in GBM tissues with CIBERSORT method (Figure 7(d)). Heat map showed the marked correlations between tumor-infiltrating lymphocytes across GBM (Figure 7(e)). Compared with the low-risk group, macrophage M2, mast cell activated, monocyte, neutrophil, NK cell resting, and T cells CD8 displayed significantly increased infiltration levels in the high-risk group (Figures 7(f) and 7(g)). In contrast, markedly reduced abundance of mast cell resting, NK cell activated, T cell CD4 memory resting, and T cell follicular helper was found in high- than low-risk groups.

### 3.8. Hypoxia-Derived Risk Score Can Predict Immune Response and Chemotherapeutic Sensitivity

Cancer-immunity cycle represents a series of functional stepwise events for obtaining an effective control of cancer growth through the immune system [29]. We quantified the activation of seven steps in cancer immunity cycle across GBM patients. As a result, each step prominently displayed higher activation in the high-risk group than the low-risk group (Figures 8(a) and 8(b)). We observed that high-risk samples exhibited markedly increased mRNA expression of immune checkpoints (TNFSF14, HAVCR2, CD209, CD226, CD274, and CD96) compared with low-risk samples (Figure 8(c)). Meanwhile, the above immune checkpoints were positively correlated to hypoxia-derived risk score (Figure 8(d)). In Figure 8(e), there was significantly higher mRNA expression of HLA-DOA, HLA-DQA1, HLA-DQB1, HLA-DRB1, HLA-DMA, HLA-DRA, HLA-DPB1, HLA-DRB6, HLA-DQA2, HLA-DPA1, HLA-DMB, HLA-DRB5, HLA-DQB2, HLA-B, and HLA-E in high- than low-risk samples. Also, most of HLA genes displayed positive correlations to hypoxia-derived risk score (Figure 8(f)). IPS score was quantified in each GBM sample. Compared with the low-risk group, increased IPS score was found in the high-risk group, indicating that high-risk patients might respond to anti-CTLA-4 or anti-PD-1 therapy (Figure 8(g)). In Figure 8(h), we observed the prominently increased TIDE score in the high-risk group in comparison to the low-risk group. We compared IC50 values of chemotherapeutic agents between high- and low-risk groups. As a result, the high-risk group displayed significantly increased IC50 values of JNK inhibitor VIII, QS11, EHT 1864, and axitinib, indicative of reduced responses to the above therapeutic agents. In contrast, the high-risk group had markedly reduced IC50 values of erlotinib, PHA 665752, dasatinib, BMS 536924, DMOG, CGP 082996, CI 1040, AZD6482, bryostatin 1, FTI 277, CGP 60474, and LFM A13, indicative of higher sensitivity to above drugs (Figure 8(i)). Collectively, hypoxia-derived risk score possessed the potential to predict immune response as well as chemotherapeutic sensitivity.

### 3.9. Genetic Mutation Landscape in High- and Low-Risk GBM

We compared the differences in genetic mutation between high- and low-risk GBM patients in TCGA dataset. Higher mutation frequency was found in the low-risk group (94.67%) than the high-risk group (88.75%). The top ten mutation genes were visualized, as shown in Figures 9(a) and 9(b). Missense mutation was the most frequent mutation type both in high- and low-risk groups (Figures 9(c) and 9(d)). There was a marked difference in EGFR mutation between two groups (Figure 9(e)). We also calculated the ore in each GBM specimen, with a median TMB of 0.86/MB (Figure 9(f)). As depicted in Figure 9(g), the low-risk group exhibited relatively higher TMB score than the high-risk group.

### 3.10. Verification of ALDH3B1 and CTSZ in GBM

ALDH3B1 and CTSZ expression was verified in human glioma cell lines (U251, SHG-44, and U87) as well as healthy glial cell line HEB via RT-qPCR and western blotting. Compared with HEB cell, ALDH3B1 and CTSZ displayed markedly higher mRNA expression in U251, SHG-44, and U87 cells (Figures 10(a) and 10(b)). Meanwhile, we observed their upregulation in glioma cells than normal glial cells (Figures 10(c)–10(e)).

## 4. Discussion

Hypoxia represents a common characteristic found in most solid tumors including GBM [30]. It possesses a wide-ranging influence on distinct biological functions such as prognosis and resistance [31]. In solid tumors, interplay between hypoxia and hallmarks of cancer induces aggressive phenotypes and resistance, eventually causing therapy failure as well as unfavorable survival outcomes [32,33]. Currently, several hypoxic genetic models have been conducted upon prognostic prediction in diverse cancers [34–36]. Nevertheless, considering that hypoxia is a complex process involving modulation networks of various genes, this study conducted a hypoxia-derived gene signature in predicting clinical outcomes of GBM patients.

Herein, we retrospectively curated the transcriptome profiling and clinicopathological characteristics of GBM from TCGA and CGGA cohorts. Among hallmarks of cancer, hypoxia represented a prominent risk factor of GBM outcomes. Through WGCNA method, we identified 271 hypoxia-derived genes. Among them, 23 genes were in relation to GBM prognosis. Afterwards, a robust hypoxia-derived gene signature was developed with LASSO method. The excellent prediction ability was confirmed across GBM. This risk score displayed a prominent advantage in predicting long-term prognosis in comparison to conventional clinical parameters. Enriched pathways were compared between high- and low-risk groups. As a result, high risk score had marked associations with aggressive molecular alterations such as angiogenesis and EMT. Based on aforementioned evidence, intratumoral hypoxia served as the major cancer hallmark and was correlated to unfavorable prognosis in GBM patients.

Immunosuppressive microenvironment presents defining biological characteristics of GBM, with many interrelated barriers that hinder effective antitumor responses [37]. The hypoxic microenvironment may recruit immunosuppressive cells, such as tumor-associated macrophage and myeloid-derived suppressor cell as well as Treg. Our data showed that hypoxia-derived gene signature possessed significant associations with cancer immunity. High risk score was predictive of higher responses to immunotherapy. Moreover, hypoxia-derived gene signature retained the prognostic capacity in discriminating high-risk populations, which might benefit from adjuvant chemotherapy. We observed that high-risk patients had higher sensitivity to erlotinib, PHA 665752, dasatinib, BMS 536924, DMOG, CGP 082996, CI 1040, AZD6482, bryostatin 1, FTI 277, CGP 60474, and LFM A13.

This hypoxia-derived gene signature contained ALDH3B1 and CTSZ that displayed prominent upregulation in GBM. ALDH3B1 is in relation to tumor size, and histological grade of lung adenocarcinoma as well as its upregulation is predictive of undesirable survival outcomes [38]. Moreover, following balancing the baseline features through propensity score matching, ALDH3B1 acts as an independent risk factor of lung adenocarcinoma outcomes. CTSZ may classify high- and low-risk glioma patients, which possesses potential prognostic potential in clinical application [39]. Our experimental evidence confirmed the upregulation of ALDH3B1 and CTSZ in GBM cells than normal glial cells. Despite this, more experiments should be utilized for investigating their biological implications in GBM progression.

Nevertheless, this retrospective study had inevitable limitations. Although we externally verified the excellent prognostic capacity of the hypoxia-derived gene signature in the CGGA dataset, this signature will be validated in a prospective cohort. Moreover, in-depth experiments will be presented for elucidating hypoxia-relevant biological implications underlying this genetic signature in GBM. Taken together, this study confirmed that hypoxia was the main risk factor for the survival of GBM patients, and at the same time, we screened effective prognostic biomarkers, which provided a theoretical basis and research direction for the precise care of GBM patients. Research on cancer hypoxia has been widely discussed. Studies have shown that oxygen inhalation, massage, heating, exercise, and other methods can effectively improve the hypoxic environment of cancer [40]. On this basis, nursing experts can incorporate hypoxia into cancer symptom nursing. The hypoxia of cancer patients, like cancer pain and cancer fatigue, should attract the attention of nursing scientists, using the Nursing Science Precision Health (NSPH) Model. Through the screening of hypoxia biomarkers, personalized and precise nursing services can be accurately carried out for high-risk groups, and the prognosis of patients can be improved. The development of bioinformatics also provides strong theoretical support for precise symptom care of cancer patients. Future nursing experts should increase the promotion and use of data science.

## 5. Conclusion

Collectively, our findings demonstrated that hypoxia acted as a prominent risk factor of GBM survival outcomes. Through integrated bioinformatic and machine learning analysis, we built a hypoxia-derived gene signature in the prediction of prognosis, recurrence, and progression as well as immuno- and chemotherapeutic responses for GBM patients. These data may offer useful clues for improving personalized management of GBM.

## Figures and Tables

**Figure 1:** Hypoxia acts as a dominant risk factor for GBM prognosis in TCGA dataset. (a) Heat map depicted the associations between hallmarks of cancer across GBM samples. Red meant positive correlation while blue meant negative correlation. (b) Heat map visualized the activation of hallmarks of cancer across GBM tissues. (c) Univariate cox regression analysis showed the associations of hallmarks of cancer with GBM prognosis. (d) Kaplan-Meier curves of OS were presented between high and low *Z*-score of hypoxia groups. (e) Sample dendrogram and trait heat map across GBM samples. (f) Identification of soft threshold (power) value according to scale independence and mean connectivity. (g) Gene dendrogram and identification of coexpression modules identified by unique colors. (h) Heat map showed the associations of coexpression module with hypoxia. (i) Gene significance across different coexpression modules.

**Figure 2:** Development of a hypoxia-derived risk score for GBM prognosis in TCGA dataset. (a) LASSO regression results with the minimum lambda of 0.1273. (b) LASSO regression profiles. (c) Univariate cox regression analysis was presented for the associations of candidate variables with GBM prognosis. (d) Heat map visualized the expression of candidate variables ALDH3B1 and CTSZ in high- and low-risk patients. (e, f) The mRNA expression of ALDH3B1 and CTSZ was compared in GBM and normal tissues. (g) Distribution of risk score across GBM patients. GBM patients were clustered into high- and low-risk groups in line with the median value. (h) Distribution of alive and dead status in high- and low-risk groups. (i) Distribution of disease-free and recurrence/progression in high- and low-risk groups.

**Figure 3:** Hypoxia-derived risk score predicts GBM prognosis, recurrence, and progression in TCGA dataset. (a–c) Kaplan-Meier curves of OS were depicted between high- and low-risk groups in the training set, testing set, and entire set. (d–f) ROC curves of 6-year survival were conducted for estimating the prediction ability of this risk score for GBM prognosis in the training set, testing set, and entire set. (g–i) Kaplan-Meier curves were utilized for comparing the differences in DFS, FSS, and PFS between high- and low-risk groups in TCGA dataset.

**Figure 4:** Hypoxia-derived risk score acts as a robust and independent risk factor for GBM prognosis. (a) Kaplan-Meier curves were conducted for externally verifying the difference in OS between high- and low-risk groups in CGGA dataset. (b) ROC curves of 3-, 4-, and 5-year survival were depicted for assessment of the predictive performance for GBM prognosis in the CGGA dataset. (c) Time-independent ROC curves were established for hypoxia-derived risk score, age, sex, and tumor purity in TCGA dataset. (d, e) Uni- and multivariate cox regression analysis was adopted for evaluating the associations of hypoxia-derived risk score, age, sex, and tumor purity with GBM prognosis in TCGA dataset. (f) Correlation between hypoxia-derived risk score and age across GBM patients was presented in TCGA dataset. (g) Hypoxia-derived risk score was compared in female and male patients in TCGA dataset. (h) Association of hypoxia-derived risk score with tumor purity was carried out in TCGA dataset. (i–k) Kaplan-Meier curves were conducted for assessing the OS differences in each subgroup stratified by hypoxia-derived risk score, age, sex, and tumor purity (TMP) in TCGA dataset.

**Figure 5:** Construction of a prognostic nomogram for GBM in TCGA dataset. (a, b) Uni- and multivariate cox regression analysis was presented for investigating the associations of hypoxia-derived risk score, age, and sex with GBM prognosis in TCGA dataset. (c) A prognostic nomogram was conducted through hypoxia-derived risk score and age in TCGA dataset. (d) Kaplan-Meier curves were depicted for OS in high and low nomogram risk groups in TCGA dataset. (e) ROC curve of 6 years was established for evaluating the predictive efficacy of this nomogram in TCGA dataset. (f) Kaplan-Meier curves of OS were conducted in high and low nomogram risk groups in the CGGA dataset. (g) ROC curve of 6 years was constructed for validating the predictive performance of the nomogram in the CGGA dataset. (h) Calibration curve was utilized for observing the nomogram-estimated and actual OS in TCGA dataset. (i) DCA was conducted for clinical benefit based on the nomogram in TCGA dataset.

**Figure 6:** Association of hypoxia-derived risk score with hallmarks of cancer in TCGA dataset. (a) GSEA results showed the first six hallmarks of cancer involved in hypoxia-derived risk score. (b) Heat map visualized the activation of hallmarks of cancer in high- and low-risk groups. (c) The activation of hallmarks of cancer was compared in two groups. ^∗^*P* < 0.05; ^∗∗^*P* < 0.01; ^∗∗∗^*P* < 0.001.

**Figure 7:** Association of hypoxia-derived risk score with tumor microenvironment of GBM in TCGA dataset. (a–c) Immune score, stromal score, and ESTIMATE score were compared between high- and low-risk groups. (d) Landscape of the abundance of tumor-infiltrating lymphocytes across GBM tissues. The color of the box indicated the correlation coefficient *R*. The darker the color, the stronger the correlation. Red represented positive correlation, and blue represented negative correlation. The number in the box represented the *P* value. “0” meant *P* < 0.001. (e) Heat map showed the correlations between tumor-infiltrating lymphocytes across GBM tissues. Red meant positive correlation while blue meant negative correlation. (f) Heat map visualized the abundance of tumor-infiltrating lymphocytes in each GBM specimen. (g) The abundance of tumor-infiltrating lymphocytes was compared between high- and low-risk groups.

**Figure 8:** Hypoxia-derived risk score can predict immune response and chemotherapeutic sensitivity across GBM patients in TCGA dataset. (a) Heat map visualized the activation of each step in cancer immunity cycle in high- and low-risk GBM groups. (b) The activation of each step in cancer immune cycle was compared in high- and low-risk GBM groups. ^∗^*P* < 0.05; ^∗∗^*P* < 0.01; ^∗∗∗^*P* < 0.001. (c) The mRNA expression of immune checkpoints was compared between high- and low-risk GBM groups. (d) Correlation of each immune checkpoint with risk score was calculated across GBM patients. (e) The mRNA expression of HLA genes was compared between high- and low-risk GBM groups. (f) Correlation of each HLA gene with risk score was calculated across GBM patients. (g) Heat map visualized the IPS score in high- and low-risk GBM groups. (h) TIDE score was compared between high- and low-risk GBM groups. (i) IC50 values of chemotherapeutic agents were compared between high- and low-risk GBM groups.

**Figure 9:** Genetic mutation landscape in high- and low-risk GBM. (a, b) The frequency of the top ten mutation genes in high- and low-risk GBM groups. Mutation type was identified by unique color. (c) Landscape of genetic mutation in the high-risk GBM group. (d) Landscape of genetic mutation in the low-risk GBM group. (e) Comparison of the first eight mutation genes between high- and low-risk GBM groups. ^∗^*P* < 0.05. (f) Distribution of TMB score across GBM samples. (g) Comparison of TMB score between high- and low-risk GBM groups.

**Figure 10:** Verification of ALDH3B1 and CTSZ in GBM. (a, b) RT-qPCR was utilized for examining the mRNA expression of ALDH3B1 and CTSZ in human glioma cell lines (U251, SHG-44, and U87) as well as healthy glial cell line HEB. (c–e) Western blotting was presented for detecting the mRNA expression of ALDH3B1 and CTSZ in human glioma cell lines (U251, SHG-44, and U87) as well as healthy glial cell line HEB. ^∗∗^*P* < 0.01; ∗∗∗∗*P* < 0.0001.

**Table 1:** Clinical features of GBM patients in TCGA dataset.

Variables	Total GBM (*N* = 160)	Training cohort (*N* = 80)	Testing cohort (*N* = 80)
Age	59.41 ± 13.62	59.74 ± 11.5	59.08 ± 15.52
Status			
Alive	31 (19.38)	19 (23.75)	12 (15)
Dead	129 (80.62)	61 (76.25)	68 (85)
Sex			
Male	104 (65)	49 (61.25)	55 (68.75)
Female	56 (35)	31 (38.75)	25 (31.25)

**Table 2:** Univariate cox regression and ROC analysis of genes in the hypoxia-related module across GBM patients in TCGA dataset.

			AUC				
Gene	*P* value	HR	3 years	4 years	5 years	6 years	7 years
CTSZ	0.001401	1.001996	0.541868	0.531175	0.519589	0.70724	0.70724
IL4I1	0.003412	1.043224	0.599506	0.519613	0.466411	0.582664	0.582664
P2RY6	0.004204	1.076029	0.415884	0.389919	0.394214	0.295217	0.295217
ALDH3B1	0.004547	1.020909	0.581294	0.60466	0.668369	0.8329	0.8329
SERPINA1	0.006526	1.002752	0.597413	0.562337	0.556287	0.677964	0.677964
CTSC	0.009301	1.002576	0.503505	0.493347	0.480802	0.576349	0.576349
OSCAR	0.011524	1.040114	0.508397	0.410077	0.503492	0.577863	0.577863
RAC2	0.011789	1.019221	0.551351	0.436907	0.345869	0.451122	0.451122
PTPN7	0.01985	1.047849	0.594861	0.581799	0.528553	0.801346	0.801346
DOK3	0.019975	1.017264	0.566994	0.611672	0.483944	0.664192	0.664192
FCGR2A	0.02197	1.002868	0.644756	0.503723	0.55335	0.742644	0.742644
NCF2	0.02279	1.012677	0.562694	0.454037	0.535923	0.609302	0.609302
APOBR	0.025558	1.036254	0.531441	0.574135	0.629578	0.885046	0.885046
SPP1	0.030952	1.000044	0.581509	0.308017	0.164882	0.188879	0.188879
NOD2	0.033034	1.051209	0.617333	0.696306	0.666013	0.566436	0.566436
DENND2D	0.034141	1.02575	0.569936	0.422816	0.401108	0.495169	0.495169
TYMP	0.036372	1.005606	0.599976	0.543437	0.613858	0.827708	0.827708
HMOX1	0.03984	1.000692	0.49011	0.418883	0.242794	0.263565	0.263565
DAB2	0.042431	1.004009	0.496005	0.448426	0.503731	0.644549	0.644549
FPR3	0.044063	1.010057	0.566919	0.414651	0.405434	0.526891	0.526891
FGR	0.045493	1.017681	0.632235	0.47959	0.595887	0.70649	0.70649
CD180	0.049196	1.023759	0.485978	0.302002	0.326194	0.362863	0.362863
FBP1	0.049958	1.020177	0.656886	0.511191	0.47078	0.518965	0.518965

Abbreviations: HR: hazard ratio; AUC: area under the curve.

## Data Availability

The datasets analyzed during the current study are available from the corresponding author on reasonable request.

## Abbreviations

GBM: Glioblastoma multiforme
TCGA: The Cancer Genome Atlas
MAF: Mutation Annotation Format
CGGA: Chinese Glioma Genome Atlas
MSigDB: Molecular Signatures Database
ssGSEA: Single-sample gene set enrichment analysis
GSVA: Gene set variation analysis
WGCNA: Weighted gene coexpression network analysis
LASSO: Least absolute shrinkage and selection operator
OS: Overall survival
DFS: Disease-free survival
DSS: Disease-specific survival
PFS: Progression-free survival
ROC: Receiver operator characteristic
DCA: Decision curve analysis
GSEA: Gene set enrichment analysis
ESTIMATE: Estimation of STromal and Immune cells in MAlignant Tumours using Expression data
CIBERSORT: Cell type Identification By Estimating Relative Subsets Of RNA Transcripts
IPS: Immunophenoscore
TIDE: T cell dysfunction and exclusion
TMB: Tumor mutation burden
HLA: Human leukocyte antigen
CGP: Cancer Genome Project
IC50: Half-maximal inhibitory concentration
HR: Hazard ratio
AUC: Area under the curve
RT-qPCR: Real-time quantitative reverse transcription PCR.
